The article "Identification of the Immune Status of Hypertrophic Cardiomyopathy by Integrated Analysis of Bulk- and Single-Cell RNA Sequencing Data" was retracted in 2023. Reasons: signs of a paper mill; compromised peer review; unreliable results or conclusions.

# Identification of the Immune Status of Hypertrophic Cardiomyopathy by Integrated Analysis of Bulk- and Single-Cell RNA Sequencing Data

**DOI:** 10.1155/2022/7153491

**Published:** 2022-10-04

**Authors:** Wei Zhao, Tianyu Wu, Jian Zhan, Zishuang Dong

**Affiliations:** ^1^Division of Cardiology, The First Affiliated Hospital with Nanjing Medical University, Nanjing 210000, China; ^2^Department of Cardiology, Xuzhou Central Hospital, Xuzhou, Jiangsu 221000, China

## Abstract

**Objectives:**

Hypertrophic cardiomyopathy (HCM) is the most common hereditary cardiomyopathy and immune infiltration is considered an indispensable factor involved in its pathogenesis. In this study, we attempted to combine bulk sequencing and single-cell sequencing to map the immune infiltration-related genes in hypertrophic cardiomyopathy.

**Methods:**

The GSE36961, GSE160997, and GSE122930 datasets were obtained from the Gene Expression Omnibus database. The compositional patterns of the 18 types of immune cell fraction and pathway enrichment score in control and HCM patients were estimated based on the GSE36961 cohort using xCell algorithm. The Weighted Gene Coexpression Network Analysis (WGCNA) was performed to identify genes associated with immune infiltration for hypertrophic cardiomyopathy. The area under the curve (AUC) value was obtained and used to evaluate the discriminatory ability of common immune-related DEGs. “NetworkAnalyst” platform was used to identify TF-gene and TF-miRNA interaction with identified common genes. Heat map was used to determine the association between common DEGs and various immune cells.

**Results:**

Immune infiltration analysis by the xCell algorithm showed a higher level of CD8+ naive T cells, CD8+ T cells, as well as a lower level of activated dendritic cells (aDC), dendritic cells (DC), immature dendritic cells (iDC), conventional dendritic cells (cDC), macrophages, M1 macrophages, monocytes, and NKT cell in HCM compared with the control group in GSE36961 dataset. aDC, macrophages, and M1 macrophages were the top three discriminators between HCM and control groups with the area under the curve (AUC) of 0.907, 0.867, and 0.941. WGCNA analysis showed that 1258 immune-related genes were included in four different modules. Of these modules, the turquoise module showed a pivotal correlation with HCM. 13 common immune-related DEGs were found by intersecting common DEGs in GSE36961 and GSE160997 datasets with genes from the genes in turquoise module. 5 hub immune-related genes (S100A9, TYROBP, FCER1G, CD14, and S100A8) were identified by protein interaction network. Through analysis of single-cell sequencing data, S100a9, TYROBP, FCER1G, and S100a8 were mainly expressed by infiltrated M1 proinflammatory cells, especially Ccr2-M1 proinflammatory macrophage cells in the heart immune microenvironment while Cd14 was expressed by infiltrated M1 proinflammatory macrophage cells and M2 macrophages in transverse aortic constriction (TAC) mice at 1 week. Higher M2 macrophage and M1 proinflammatory macrophage infiltration as well as lower Ccr2-M1 proinflammatory macrophage and dendritic cells were shown in TAC 1week mice compared with sham mice.

The article "Identification of the Immune Status of Hypertrophic Cardiomyopathy by Integrated Analysis of Bulk- and Single-Cell RNA Sequencing Data" was retracted in 2023. Reasons: signs of a paper mill; compromised peer review; unreliable results or conclusions.

**Conclusions:**

There was a difference in immune infiltration between HCM patients and normal groups. aDC, macrophages, and M1 macrophages were the top three discriminator immune cell subsets between HCM and control groups. S100A9, TYROBP, FCER1G, CD14, and S100A8 were identified as potential biomarkers to discriminate HCM from the control group. S100a9, TYROBP, FCER1G, and S100a8 were mainly expressed by infiltrated M1 proinflammatory cells, especially Ccr2-M1 proinflammatory cells in the heart immune microenvironment while Cd14 was expressed by M2 macrophages in transverse aortic constriction (TAC) mice at 1 week.

## 1. Introduction

Hypertrophic cardiomyopathy is the most common genetic cardiomyopathy [1]. Clinical manifestations vary widely and can lead to sudden cardiac death in severe cases [2]. Current symptomatic treatments can only delay the progression of the disease, but they cannot reverse it [3]. Previous studies have shown that mutations in some genes involved in encoding sarcomere are directly associated with HCM [4].

The heart is a complex multicellular organ composed of cardiomyocytes, fibrocytes, immune cells, and endothelial cells. More and more studies have shown that immune cells play a role in the pathogenesis of the cardiovascular disease, including hypertrophic cardiomyopathy [5]. Many studies have shown that immune cells are involved in the regulation of cardiac homeostasis and physiological and pathological processes [6]. Meanwhile, cellular communication between immune cells and other cardiac constituent cells plays an important role in the composition of hypertrophic cardiomyopathy [7]. xCell algorithm is an algorithm to identify the abundance of immune infiltrates in tissues based on transcriptome data, which has been widely used to characterize the immune microenvironment of tumors and immune diseases [8].

Through single-cell sequencing (scRNA-seq), researchers can further examine gene expression in individual cells and attempt to locate functional differences between different clinical phenotypes, particularly immune cells [9, 10]. The characteristics of immune microenvironment in hypertrophic cardiomyopathy are limited, so in this study, to describe the immune cells in hypertrophic cardiomyopathy, we combined conventional sequencing data of human hypertrophic cardiomyopathy with scRNA-seq data from transverse aortic constriction (TAC) model. This can be better used to explore and understand functional cell clusters associated with hypertrophic cardiomyopathy.

The article "Identification of the Immune Status of Hypertrophic Cardiomyopathy by Integrated Analysis of Bulk- and Single-Cell RNA Sequencing Data" was retracted in 2023. Reasons: signs of a paper mill; compromised peer review; unreliable results or conclusions.

## 2. Methods

### 2.1. Data Collection

Two gene expression profile datasets (GSE36961 and GSE160997 datasets) were downloaded from GEO database. GSE36961 contains surgical myectomy tissue from 106 HCM patients and 39 control patients. Samples for GSE160997 were obtained from the anterior septal tissues of 18 HCM patients and 5 control patients. The expression value was preprocessed using the “normalize between arrays” function in the “limma” package. The list of immune-related genes was downloaded from the ImmPort database.

### 2.2. Immune Cell Infiltration Analysis

Correlation matrix of immune cell subtypes and hub genes was constructed by “corrplot” in R. Pearson correlation coefficients were calculated and used for evaluating the strength of correlation.

### 2.3. ROC Analysis of DEGs

We conducted DEG analysis with normalized expression data using “limma” R package [11] (abs(logFC) > 1 and adjusted *P*value < 0.05). To evaluate the diagnostic value of DEGs, ROC analysis was conducted.

### 2.4. Calculate Enrichment Scores of Immune-Related Pathways

The pathway enrichment score was calculated based on the single-sample gene-set enrichment analysis (ssGSEA) using the immune-related gene set to quantify the expression levels of these genes for each HCM and control patients [12].

### 2.5. Biological Enrichment Analysis

The biological function for DEGs was analyzed by Gene Ontology (GO) enrichment analysis using the R package “clusterProfiler” [13].

### 2.6. Summarize the Expression Levels of Immune-Related DEGs from Single Cell Sequence Data of Human Protein Atlas (HPA) Database

HPA database [14] was used to find the expression of immune-related DEGs in each type of cells in heart tissues, and the relative expression ratio of genes in each immune cell was obtained by stacking histogram.

### 2.7. Single-Cell Data Processing

Raw data for GSE122930 were downloaded from the portal website, and the package of Seurat was used to process data [15]. The raw data GSE122930 contains one sample for sham 1-week mice, two samples for sham 4-week mice, two samples for TAC 1-week mice, and two samples for TAC 4-week mice. For B cell cluster, signatures of Cd79a, Cd79b, and Cd19 were chosen for annotation. For activated B cell, signatures of Cd86, Cd69, and Cxcr5 were chosen for annotation. For T cell cluster, signatures of Tcf7, Cd8b1, Cd8a, and Thy1 were chosen for annotation. For regulatory T cell cluster, signatures of Pdcd1 and Ctla4 were chosen. For activated T cell cluster, signatures of Cd69 and Ccr7 were chosen for annotation. For monocyte and macrophage cluster, signatures of Cd14, Cd68, Ccr2, and Adgre1 were chosen for annotation. For M2 macrophage cluster, signatures of Cd163 and Mrc1 were chosen for annotation. For M1 proinflammatory macrophage cluster, signatures of Il1b were chosen for annotation. For dendritic cell cluster, signatures of Cd209a were chosen for annotation. For neutrophil cluster, signatures of Cd209a were chosen for annotation. For mast cell cluster, signatures of Mcpt8 and Il6 were chosen for annotation. For NK cell cluster, signatures of Gzma, Ncr1, and Klrb1c were chosen for annotation.

The article "Identification of the Immune Status of Hypertrophic Cardiomyopathy by Integrated Analysis of Bulk- and Single-Cell RNA Sequencing Data" was retracted in 2023. Reasons: signs of a paper mill; compromised peer review; unreliable results or conclusions.

## 3. Results

### 3.1. Immune Cell Landscape of Heart Tissue Transcriptome between HCM Patients and Control

Cardiac tissue transcriptome from 106 HCM patients and 39 control in GSE36961 dataset were included in the study. xCell algorithm was performed to analyze immune cell fractions among these two groups. Immune infiltration analysis by the xCell algorithm showed a higher level of CD8+ naive T cells, CD8+ T cells, as well as a lower level of activated dendritic cells (aDC), dendritic cells (DC), immature dendritic cells (iDC), conventional dendritic cells (cDC), macrophages, M1 macrophages, monocytes, and NKT cell in HCM compared with the control group in GSE36961 dataset (Figure 1(a)). The total immune cell score gained by the xCell algorithm showed that HCM had a significantly lower immune cell score than the control. aDC, macrophages, and M1 macrophages were the top three discriminators between HCM and control groups with the area under the curve (AUC) of 0.907, 0.867, and 0.941 in GSE36961 dataset (Figure 1(b)). These three immune cell subsets all got an AUC of 1.000 in GSE160997 dataset. Proportions of immune cell subsets in HCM and normal groups were detailed in Figure 1(c). Total immune cell scores showed immune cell scores of HCM patients were significantly lower than control (Figure 1(d)). Pathway enrichment analysis by ssGSEA showed a lower score for antigen processing and presentation pathway, antimicrobial pathway, BCR signaling pathway, chemokine receptor pathway, cytokine receptor pathway, cytokine pathway, interleukin pathway, interleukin receptor pathway, natural killer cell cytotoxicity pathway, TCR signaling pathway, TGF-*β* family member pathway, TGF-*β* family member receptor pathway, TNF family member pathway, and TNF family member receptor pathway in HCM compared with the control group (Figure 1(e)). These results indicated that the infiltration of immune cells in the heart tissue of HCM patients was significantly lower than normal and the activation of immune pathways was low.

The article "Identification of the Immune Status of Hypertrophic Cardiomyopathy by Integrated Analysis of Bulk- and Single-Cell RNA Sequencing Data" was retracted in 2023. Reasons: signs of a paper mill; compromised peer review; unreliable results or conclusions.

### 3.2. Construction of Weighted Coexpression Network Based on 1258 Immune-Related Gene Transcriptome and Identification of Key Module for HCM

1258 immune-related genes were downloaded from ImmPort database. A weighted coexpression network was constructed and four modules were identified (Figure 2(a)). There were 219 genes in the blue module, 31 genes in the brown module, 610 genes in the grey module, and 398 genes in the turquoise module. The 398 immune-related genes in the turquoise module had a significant negative correlation with HCM and the correlation coefficient is −0.83 (Figure 2(b)). The relationship between different modules was shown in Figure 2(c). The correlation between gene module membership value in the turquoise module and gene significance value for HCM is visualized in Figure 2(d).

### 3.3. Identification of 5 Hub Immune-Related DEGs for HCM

GO and KEGG enrichment analysis found that 398 genes in the turquoise module are mainly involved in natural killer cell-mediated cytotoxicity, cytokine-cytokine receptor interaction, cytokine activity, and cytokine receptor binding (Figure 3(a)), which indicated immune response is involved in the pathogenesis of HCM. A total of 128 DEGs between HCM and control were obtained; 38 genes were significantly upregulated and 90 genes were significantly downregulated (abs(logFC) > 1 and adjust *P*value < 0.05) (Figure 3(b)). 13 common immune-related DEGs were found by intersecting common DEGs in GSE36961 and GSE160997 datasets with genes from the genes in turquoise module (Figure 3(c)). Correlation heat map between 13 common immune-related DEGs was shown in Figure 3(d). 5 hub immune-related genes (S100A9, TYROBP, FCER1G, CD14, and S100A8) were identified by the protein interaction network (Figure 3(e)). All hub immune-related genes were significantly downregulated in HCM.

### 3.4. Predictive Performance of Five Hub Immune-Related DEGs for HCM

The single-cell data of normal heart tissue in the Human Protein Atlas (HPA) database indicated S100A8, S100A9, TYROBP, CD14, and FCER1G are mostly expressed in the immune cells of heart tissue (Figure 4(a)). S100A9 was identified as the best potential biomarker with an area under the ROC curve (AUC) of 0.963 in the GSE36961 dataset (Figure 4(b)), while FCER1G was identified as the best potential biomarker with an area under the ROC curve (AUC) of 1.000 in the GSE160997 dataset (Figure 4(c)). TF-gene interactions and TF-miRNA coregulatory network were collected using “NetworkAnalyst” for five hub immune-related DEGs. SPl1, FLl1, RUNX1, and TFAP2C were the top four transcription factors by the TF-gene network (Figure 4(d)) while hsa-miR-196a was the top microRNA that may regulate the expression of core immune-related genes (Figure 4(e)).

The article "Identification of the Immune Status of Hypertrophic Cardiomyopathy by Integrated Analysis of Bulk- and Single-Cell RNA Sequencing Data" was retracted in 2023. Reasons: signs of a paper mill; compromised peer review; unreliable results or conclusions.

### 3.5. Further Demonstration of Immune Microenvironment and Hub Immune-Related Genes in TAC 1 w Mice

In addition to bulk sequencing analysis, we analyzed the immune microenvironment of TAC 1 w mice with single-cell sequencing dataset GSE122930. We simulated HCM in mice with transverse aortic coarctation for 1 week. We further clustered immune cell populations into 13 clusters and using genes Cd79a, Cd79b, Cd19, Cd86, Cd69, Cxcr5, Pdcd1, Ctla4, Cd69, Ccr7, Cd163, Mrc1, Il1b, Cd209a, Mcpt8, Il6, Gzma, Ncr1, and Klrb1c, we classified 13 cell clusters into 10 cell populations, which were B cell, activated B cell, activated T cell, regulatory T cell, M2 macrophage, M1 proinflammatory macrophage, Ccr2-M1 proinflammatory macrophage, dendritic cell, mast cell, and NK cell (Figure 5(a)). Higher M2 macrophage and M1 proinflammatory macrophage infiltration as well as lower Ccr2-M1 proinflammatory macrophage and dendritic cells were shown in TAC 1week mice compared with sham 1week mice (Figure 5(b)). S100a9, TYROBP, FCER1G, and S100a8 were mainly expressed by infiltrated M1 proinflammatory cells, especially Ccr2-M1 proinflammatory cells in the heart immune microenvironment while Cd14 was expressed by M1 proinflammatory cells and M2 macrophages in transverse aortic constriction (TAC) mice at 1 week (Figures 5(c) and 5(d)).

### 3.6. Hub Immune-Related Genes Were Downregulated in Ccr2-M1 Proinflammatory Macrophage and a High Correlation Were Found between Hub Immune-Related Genes and M1 Proinflammatory Macrophage Markers in Bulk Sequencing Data

All five hub genes (S100a9, TYROBP, FCER1G, S100a8, and Cd14) were significantly downregulated in Ccr2-M1 proinflammatory macrophage between TAC 1week mice and sham 1week mice (Figures 6(a)–6(e)), which is consistent with the changes between HCM patients and control group by bulk sequencing analysis. We further examined the correlations between hub immune genes and scores for M1 macrophage cell infiltration in GSE36961 dataset, calculated by xCell methods, and the results showed hub immune genes were highly correlated with M1 macrophage cells (Figure 6(f)). We further used database GSE36961 to examine M1 macrophage cell markers' correlation with hub immune genes, and results showed hub immune genes were highly correlated with IL1B and OSM in bulk sequencing data of HCM (*P*value < 0.01) (Figure 6(g)).

## 4. Discussion

Hypertrophic cardiomyopathy is a serious hereditary cardiomyopathy, which often causes sudden death. Many studies showed that uncommon immune activation and immune cell infiltration are associated with the occurrence of heart diseases, especially atherosclerosis, coronary heart disease, and heart failure [16]. Exploring key immune-related cell enrichment and genes associated with the immune cells in the pathogenesis of hypertrophic cardiomyopathy can elucidate the involvement and regulation of immunity in the pathogenesis of HCM to a certain extent, thus providing potential therapeutic targets for immunotherapy of hypertrophic cardiomyopathy in the future.

The article "Identification of the Immune Status of Hypertrophic Cardiomyopathy by Integrated Analysis of Bulk- and Single-Cell RNA Sequencing Data" was retracted in 2023. Reasons: signs of a paper mill; compromised peer review; unreliable results or conclusions.

More and more studies have shown that there is a close relationship between macrophages and hypertrophic cardiomyopathy [17, 18]. Macrophages are mainly divided into two subtypes, one is M1-like macrophages which may be proinflammatory, and the other is M2-like macrophages which are involved in anti-inflammatory processes in major diseases. Macrophage cells are the most important members of the heart's immune cells [19] and play an important role in maintaining homeostasis in the heart before the injury and in the repair and reconstruction of heart tissue when the heart muscle is struck. In a normal condition heart, the resident macrophages of the heart eat dead or senescent cells and maintain electrical conduction between cardiomyocytes [20]. When the heart begins to age, macrophages convert from M2-like macrophages to M1-like macrophages and promote the process of cardiac aging [21]. When cardiomyocyte necrosis occurs, bone marrow and circulating macrophages are mobilized and gathered to the infarct place and produce a variety of mediators (many kinds of chemokines, cytokines, and matrix metalloproteinases which promote collagen production and growth-promoting factors), eat damage cells, and promote angiogenesis of necrotic myocardium and scar reconstruction [22]. Considering that macrophages are important in both the physiological and pathological states of cardiovascular disease, studying the dynamics of macrophages can help us understand the role of macrophages in hypertrophic cardiomyopathy.

The Ccl2 chemokine mediates the outflow of monocytes beginning in the pool of bone marrow and gathering into inflammatory areas by combining with the receptor of Ccr2 chemokine. Macrophages derived from Ccr2-KO bone marrow mice showed polarization to M1-like macrophages from transcriptomic analysis and higher production of proinflammatory cytokines (IL6, TNF-*α*) when treated with LPS [23]. Tissue-resident Ccr2-macrophages inhibit monocyte recruitment during cardiac injury [24]. According to the expression level of Ccr2, we defined a new M1-type macrophage: Ccr2-M1 proinflammatory macrophage. A lower proportion of Ccr2-M1 proinflammatory macrophage was found in TAC 1week mice compared with sham 1week mice, which is correlated with the changes of M1 macrophage proportion in HCM patients compared with control.

The article "Identification of the Immune Status of Hypertrophic Cardiomyopathy by Integrated Analysis of Bulk- and Single-Cell RNA Sequencing Data" was retracted in 2023. Reasons: signs of a paper mill; compromised peer review; unreliable results or conclusions.

The alarmins S100A8 and S100A9 are especially expressed by neutrophils as the inactive heterodimer S100A8/A9, also identified as calprotectin, and are quickly released to the extracellular environment when stimulated with inflammatory mediators and act as inflammation-related molecular biomarkers [25]. Neutrophils are the main cells producing S100A8/A9 [26], but the protein S100A8/A9 is also secreted by other types of cell-like endothelial cells, platelets, monocytes, and macrophages [27]. Extracellular S100A8/A9 combines with the TLR4 (Toll-like receptor 4) and RAGE (receptor of advanced glycation end products) [28, 29] and can be a potential activator for response to the innate immune system in various types of diseases with the participation of immune and inflammatory cells [30]. TYROBP is a type I transmembrane protein which is composited by a leader peptide, a cysteine residue of the extracellular region, a segment of transmembrane, and an immunoreceptor tyrosine-based activation motif (ITAM) in the cytoplasmic domain [31]. TYROBP is mainly derived from many kinds of immune cells, such as natural killer cells, macrophages, oligodendrocytes, and osteoclasts in peripheral blood, influencing immune cell function by transmitting proinflammatory or anti-inflammatory signals [32]. TYROBP is an adaptor protein containing ITAM, and it combines with various types of receptors that promote the activation of cellular response [33]. FCER1G is a gene on chromosome 1q23.3 [34]. FCER1G binds with other proteins and involves in many nuclear processes [35]. Specifically, FCER1G is involved in the construction of the interleukin 3 (IL3) receptor complex and immunoglobulin E (IgE) receptor. It is mostly involved in transferring the proinflammatory signals of immune cells, and mediating the generation of interleukin 4 (IL4) by basophils [36]. CD14 was the first pattern recognition receptor (PRR) that combines with LPS. CD14 is identified as a common receptor for many Toll-like Receptors (TLRs) which passes bacterial cell-derived protein to TLRs to activation of cellular response [37]. In addition to its functions in innate immunity, CD14 plays an important role in regulating atherosclerosis, metabolic disease, cancer, and so on. Our results further demonstrate that these hub immune-related genes may be involved in the immune process for HCM; it may associate with M1 macrophage infiltration for HCM.

In this study, we identified three cell infiltration sets (aDC, macrophages, and M1 macrophages) and five hub immune-related genes (S100A9, TYROBP, FCER1G, CD14, and S100A8) between HCM and control groups by combining single-cell and bulk sequencing technology. All hub immune-related genes were positively correlated with M1 macrophage infiltration. We speculate that the decrease in the M1 macrophages is an important immune process in HCM. Our findings were further validated on the TAC animal model as well.

The article "Identification of the Immune Status of Hypertrophic Cardiomyopathy by Integrated Analysis of Bulk- and Single-Cell RNA Sequencing Data" was retracted in 2023. Reasons: signs of a paper mill; compromised peer review; unreliable results or conclusions.

However, our study has some limitations. Firstly, our study was based on immune infiltration analysis by the xCell algorithm from the transcriptomic profiles in available datasets. Secondly, whether there is a clear relationship between immune cell infiltration and HCM cannot be determined. Finally, the TAC model is commonly used to simulate hypertrophic cardiomyopathy, but their pathogenesis differs because HCM is more inclined to genetic disease. At the same time, patients with HCM may have a disturbed systemic immune response. Therefore, the combination of peripheral blood cell single-cell RNA sequence may provide us with a more comprehensive understanding of the patient's immune status. Although there is a large amount of literature supporting the rationality of this approach, further experiments are still needed to verify it.

## 5. Conclusion

In summary, through bioinformatics analyses, three cell infiltration sets (aDC, macrophages, and M1 macrophages) and five hub immune-related genes (S100A9, TYROBP, FCER1G, CD14, and S100A8) were acted as the potential key immune cells and genes in HCM.

## Figures and Tables

**Figure 1:** (a) The differences in 18 immune cell subsets between the HCM and control group by using xCell algorithm (^∗^ means *P* < 0.05, ^∗∗^ means *P* < 0.01, ^∗∗∗^ means *P* < 0.001, and ^∗∗∗∗^ means *P* < 0.0001). (b and c) An area under the ROC curve (AUC) of three immune cell subsets (aDC, macrophages, and M1 macrophages) in the GSE36961 and GSE160997 cohorts. (d) The difference in immune cell score between the HCM and control group by *t*-test (# means *P* < 0.0001). (e) Pathway enrichment analysis by ssGSEA between control and HCM group (^∗^ means *P* < 0.05,^∗∗^ means *P* < 0.01, ^∗∗∗^ means *P* < 0.001, and ^∗∗∗∗^ means *P* < 0.0001).

**Figure 2:** (a) The cluster dendrogram of 1258 immune-related genes in GSE36961 dataset. Each branch in the figure represents one gene, and every color represents one coexpression module. (b) Heat map of the association between modules and the illness status of HCM. The turquoise module showed to be more correlated with HCM. (c) The correlation heat map plot of three modules in GSE36961 dataset. (d) By WGCNA method, we calculated module membership and gene significance score of each gene. This figure showed the relationship between module membership score in the turquoise module and gene significance score for HCM.

The article "Identification of the Immune Status of Hypertrophic Cardiomyopathy by Integrated Analysis of Bulk- and Single-Cell RNA Sequencing Data" was retracted in 2023. Reasons: signs of a paper mill; compromised peer review; unreliable results or conclusions.

**Figure 3:** (a) GO and KEGG enrichment analysis of 398 genes in turquoise module gained by WGCNA method. (b) The volcano figure of 128 differently expressed genes (DEGs) between HCM and control group. (c) Wayne figure of three gene sets (common DEGs in GSE36961, GSE160997 datasets, and genes in turquoise module). (d) Correlation analysis between 13 common immune-related DEGs. (e) PPI network of 13 common immune-related DEGs.

**Figure 4:** (a) The expression of five hub immune-related genes calculated by the single cell data of normal heart tissue in Human Protein Atlas (HPA) database. (b and c) An area under the ROC curve (AUC) of five hub immune-related genes (S100A8, S100A9, TYROBP, CD14, and FCER1G) in the GSE36961 and GSE160997 cohorts. (d) TF-gene interactions and TF-miRNA coregulatory network of five hub immune-related genes calculated by “NetworkAnalyst” platform.

**Figure 5:** (a) Cell clusters for GSE122930 of two TAC 1 w mice. (b) Portions of different cell clusters between sham 1 w mice and TAC 1 w mice. (c and d) Expression level of five hub immune-related genes in different cell clusters of TAC 1 w mice.

**Figure 6:** (a–e) Expression level of five immune-related genes in Ccr2-M1 proinflammatory macrophage between TAC 1week mice and sham 1week mice. (f and g) Correlation between hub immune genes and scores for M1 macrophage cell infiltration and M1 macrophage cell markers (IL1B and OSM) in GSE36961.

## Data Availability

The data that support the finding of this study are available from the corresponding upon reasonable request.

## Abbreviations

HCM: Hypertrophic cardiomyopathy
WGCNA: Gene coexpression network analysis
AUC: Area under the curve
ROC: Receiver operating characteristic curve
aDC: Activated dendritic cells
iDC: Immature dendritic cells
cDC: Conventional dendritic cells
TAC: Transverse aortic constriction
S100A9: S100 calcium binding protein A9
TYROBP: Transmembrane immune signaling adaptor
FCER1G: Fc epsilon receptor Ig
S100A8: S100 calcium binding protein A8
